The article "Judicial Application of Punitive Damages for Ecological Environment Infringement in Civil Public Interest Litigation" was retracted in 2023. Reasons: unreliable results or conclusions; concerns about the data; concerns about the results or conclusions; concerns about the peer review.

# Judicial Application of Punitive Damages for Ecological Environment Infringement in Civil Public Interest Litigation

**DOI:** 10.1155/2022/6127388

**Published:** 2022-09-23

**Authors:** Yuanqing Chen

**Affiliations:** School of Law, Fuyang Normal University, Fuyang 236037, China

## Abstract

This study aimed to explore the judicial application of punitive damages for ecological environment infringement in civil public interest litigation. *Methods*. Combined with a case, the judicial application of punitive damages for ecological environment infringement in civil public interest litigation was analyzed. *Results*. After thinking and judgment, the total cost of repairing the enterprise plot in the case was 2168000 yuan, the cost of environmental functional loss was 57135.45 yuan, the cost of taking relevant emergency measures such as new drinking water and laundry Wharf Engineering was 532860.11 yuan, and the cost of testing and identification was 95670 yuan. *Conclusion*. The judicial application should be fully considered in the process of civil public interest litigation to ensure that the punitive compensation for ecological environment infringement is more reasonable.

## 1. Introduction

With the high-quality development of economic construction and the continuous improvement of social living standards, the broad masses of the people have increasingly urgent needs for a green livable environment such as fresh air and clear water, and the pursuit of a beautiful natural ecology with blue sky and green trees [1]. Building a good ecological environment is the most extensive social public welfare and the most conducive to the well-being of human beings. At the 19th National Congress of the Communist Party of China, “adhering to the harmonious coexistence between man and nature” was clearly defined as the basic strategy for upholding and developing socialism with Chinese characteristics in the new era. The Fifth Plenary Session of the 19th CPC Central Committee proposed that we should adhere to the policy of clear water and beautiful mountains, respect nature, conform to nature, protect nature, and resolutely maintain ecological security borders [2]. The infringement of polluting the environment and destroying the ecology not only infringes on property rights, even the rights to life and health of ordinary people, but also causes irreparable damage to social public interests.  Figure 1 gives the composition of the sustainable development concept.

On May 28, 2020, the third session of the 13th National People's Congress voted to adopt the civil code (Figure 2), which integrates the construction of ecological civilization into the blood of social and economic construction, injects a “green growth gene” into China, establishes the principle of green development, and plays a guiding and encouraging role in saving resources and protecting the ecological environment through civil action [3, 4]. The principle of green development is implemented into specific tort liability, which is reflected in the special provisions on the liability for pollution to the social environment and damage to the ecosystem. A punitive compensation system for ecological environment infringement is added, which not only considers the rights and interests of compensation and filling in the damage but also considers punishing the infringement so as to deter and prevent similar environmental pollution and ecological destruction and protect the public interest. The ecological environment damage compensation system, which was added to the list of tort liability for the first time, made it clear that infringers who maliciously pollute the social environment and destroy the ecosystem should bear more adverse legal consequences, which increased the illegal cost of environmental pollution and ecological destruction and also increased the legal liability of malicious infringers [5]. Although supported by the system, it still needs the joint efforts of academia and industry to achieve the legislative purpose of how to solve the practical problems of high law-abiding cost and low illegal cost in the existing ecological environment infringement through the punitive compensation system and how to improve the ecological environment protection system [6, 7].

## 2. Literature Review

Public interest litigation (Figure 3) includes civil public interest litigation and administrative public interest litigation, which are divided according to the nature of the applicable procedural law or the different objects of litigation (objects). According to the theory of procedural law, if the interests are damaged, the victim has the right to sue the court and request judicial relief [8]. According to the subject of litigation, public interest litigation can be divided into public interest litigation filed by procuratorial organs and public interest litigation filed by other social groups and individuals. The former is called civil public prosecution or administrative public prosecution, and the latter is called general public interest litigation.

“Tragedy of the commons” is a well-known phenomenon in economic circles, and it is also a widespread reality. In a foreign country, someone has done an interesting experiment, taking a piece of grassland, which is divided into several pieces and distributed to shepherds, but one piece is left in the middle as public land, which can be freely used by every shepherd [9, 10]. As a result, sociologists found that over the course of a year, the grassland allocated to individuals was used in a planned and controlled manner, while the grassland used as public land was barren because of overgrazing. The experiment concludes that because everyone has the nature to expand their living space and resources, when the public interest is in a state of no management, everyone will consciously or unconsciously squeeze public resources for their own use. Therefore, the public interest without protection is the most vulnerable to infringement. According to the theory of procedural law, if the interests are damaged, the victim has the right to sue the court and request judicial relief, just as if another shepherd's sheep ate your grassland, you can ask him to compensate. However, in theory, the public grassland belongs to all shepherds. If its interests are damaged, who will file a lawsuit? With the extension of the social public sphere and the growth of the number of public affairs, people are facing such problems in the national law. Public interest litigation is a means of litigation to solve the “tragedy of the commons.” Its emergence and development in China reflects the urgent need for the protection of public interests.

As for what public interest litigation is, there is no consensus within and between the practical and theoretical circles. The procuratorial organs are mainly responsible for promoting public interest litigation in the practical departments and most of them advocate civil public prosecution (or civil prosecution) (Figure 4). In the theoretical circle, procedural law scholars have conducted independent research on the two aspects of administrative public interest litigation and civil public interest litigation and have given the definitions of civil public interest litigation and administrative public interest litigation. However, some commentators have made a relatively complete definition of public interest litigation, but in the specific discussion, they often only discuss civil public interest litigation or administrative public interest litigation of public interest litigation [11, 12].

As for the definition of public interest litigation, one kind of view refers to the activities that specific state organs and relevant organizations and individuals, according to the authorization of the law, sue to the court for violations of laws and regulations, national interests, social interests, or the interests of specific others, and the court will investigate legal responsibilities according to law [13]. This view can be called “the broad theory of relief object.” In a broad sense, another view holds that the so-called interests of others refer to “unspecified interests of others.” Corresponding to the broad sense, some people believe that public interest litigation refers to the activity that any organization and individual can, according to the authorization of laws and regulations, have the right to sue the court for violations of the law, national interests, and social public interests, and the court will investigate the legal responsibility of the violator. This view can be called “the narrow sense of the relief object.” Public interest litigation refers to the action that damages the social public interests but does not directly damage the interests of the plaintiff, so it has no direct interest with the plaintiff himself. Of course, the behavior that damages the social public interest ultimately damages the personal interests. There is a natural connection between public interests and personal interests [14, 15].

Most people believe that the subjects who can file public interest litigation include the general public, social organizations, and procuratorial organs. What is worth discussing is what conditions individuals and groups are the legitimate parties or the eligibility of the parties. From the perspective of the purpose and nature of public interest litigation, it seems that strict restrictions should not be imposed, but out of fear of excessive litigation, it is required to properly prevent and control the parties with certain standards. Because public interest litigation involves public interests, and individuals have limited ability to bear the relevant litigation burden in litigation, individuals have relatively weak enthusiasm to file public interest litigation, and organizations, especially public interest organizations, are of great significance to promote public interest litigation. Public welfare organizations are nonprofit organizations with the purpose of promoting and protecting public interests, such as consumer associations, associations of the disabled, children's protection organizations, animal protection organizations (Figure 5), and public welfare law firms. Because public welfare organizations aim to promote and protect public interests, they pay more attention to relevant public interests and can become active promoters of public interest litigation. Therefore, a group that meets the legal conditions and the purpose of its articles of association should have the litigation qualification of public interest litigation.

## 3. Ecological Environment Infringement

Ecological infringement refers to the harmful behavior carried out by multiple and multilevel ecological infringement subjects based on different degrees of understanding, which infringes on the natural survival mode and existence form of life, destroys the natural evolution process and life reproduction process of life, and has the risk of causing ecosystem imbalance or early extinction of species, as well as a factual state that leads to the actual consequences of endangering the balanced development of ecosystem [16].

First, the legal characteristics of ecological infringement (Figure 6). From the meaning of ecological infringement, we can see that ecological infringement is a special infringement form with its own legal attributes, which is different from the traditional legal form. The subject has diversity and the progressive nature of infringement ability, the object has naturalness and limitations, the subjective aspect has cognitive hierarchy, and the objective aspect has relationship complexity.

Second, the boundary scope of ecological infringement. Because ecological infringement is an extremely special form of infringement, its conceptual basis is closely related to but different from traditional civil infringement and ecological crime [17].

Third, the difference between ecological infringement and civil infringement (Figure 7). Civil tort refers to the behavior that the perpetrator should bear civil liability according to law because of his fault to infringe on others' property and personal as well as other harmful behaviors that the law stipulates should bear civil liability for the victim. Ecological infringement and civil infringement belong to the category of infringement, and the subject of the act should bear civil liability for its behavior, and this civil liability has both sanctions and compensation.

Fourth, the difference between ecological infringement and ecological crime. Ecological crime refers to a kind of harmful social behavior in which the perpetrator intentionally or negligently infringes on the natural survival mode and existing form of life, destroys the natural evolution process and life reproduction process of life, causes the risk of ecosystem imbalance (Figure 8) or early extinction of species (Figure 9), and leads to the actual consequences of endangering the balanced development of ecosystem [18].

Fifth, the imputation principle of ecological infringement. The principle of liability fixation of ecological infringement refers to the principle of confirming the civil liability of the subject according to what standard after the fact that the infringement committed by the subject of ecological infringement has caused damage to the ecological environment. The principles of ecological tort liability include the intentional liability principle, fault liability principle (Figure 10), no-fault liability principle, objective liability principle, and absolute liability principle [19].

## 4. Research Methods

### 4.1. Case Summary

A company was registered and established, and its main business scope is the production, wholesale, and sales of chemical products. In order not to affect the normal production and operation, in the case that the equipment of the company is damaged and the sodium sulfate waste liquid generated in the production process cannot be normally treated, the manager of the production department asked the legal representative for permission to hand over the sodium sulfate waste liquid to the manager without hazardous waste disposal qualification for treatment. According to the identification of the judicial identification center, sodium azide exists in the water body and surface soil at the dumping point, and the polluted surrounding environment covers about 8.08 mu. There is sodium azide pollution in the surface soil of the dumping point. The actual calculation of the two dumping points: the total cost of land restoration (a) is 2168000 yuan, the total cost of environmental functional loss (b) is 57135.45 yuan, the cost of taking relevant emergency measures such as new drinking water and laundry Wharf Engineering (c) is 532860.11 yuan, and the total cost of detection and identification (d) is 95670 yuan. The procuratorate believes that the company's illegal disposal of sodium sulfate waste liquid from production due to equipment damage has led to serious environmental pollution in two places, affecting the drinking water of more than 1000 people, destroying the natural ecology, and damaging social and public interests. Therefore, the company filed an environmental public interest lawsuit in accordance with the law, requesting a judgment to compensate the ecological environment restoration cost, environmental function loss cost, emergency disposal cost, testing fee, and identification fee totaling 2853665.56 yuan, bearing the punitive compensation for environmental pollution of 171406.35 yuan and making an apology to the public on the national news media [20].

The calculation formula is as follows:

(1) $$\begin{array}{c} \text{Total compensation}=A+B+C+D. \end{array}$$

After calculation, the formula is as follows:

(2) $$\begin{array}{c} \text{Total compensation}=2168000+57135.45+532860.11+95670. \end{array}$$

### 4.2. Court Decision

The people's court held that the company illegally disposed of sodium sulfate waste liquid after the equipment was damaged, which led to the destruction of water and soil and the pollution of the ecological environment. The waste liquid dumping site undertakes important ecological functions such as water source, which directly pollutes the environment, damages the ecological rights and interests that the people should enjoy, and meets the applicable conditions of punitive compensation for environmental infringement stipulated in article 1232 of the civil code. On January 4, 2021, the people's court made the following judgment according to law: the company compensated for the cost of ecological environment restoration, the cost of ecological environment functional loss, the cost of emergency disposal, the cost of detection and identification, and assumed punitive compensation for environmental pollution, totaling 3025071.91 yuan. The company made an apology to the public on the national news media for the consequences of polluting the ecological environment and damaging social public interests caused by the illegal dumping of sodium sulfate waste liquid.

It is reported that this is the first case in China to apply article 1232 of the civil code on punitive compensation for environmental pollution. The other environmental pollution crime involved in the case has been concluded by the court, and the company's personnel in charge of safe production, personnel without waste treatment qualifications, and personnel who specifically carried out transportation and dumping were investigated for criminal responsibility according to law. After the case was adjudicated, the company fully recognized the serious harm caused by its own mistakes; expressed sincere repentance, apology, and obedience to the judgment; said in court that it would not appeal; and said that it would immediately pay all the repair costs and punitive damages.

### 4.3. Problems and Thoughts Caused by the Case

From the perspective of legal practice, the introduction of the punitive damage system originally belonging to the common law system is not the result of theoretical evidence, but out of the need to solve practical problems, that is, it adopts problem-oriented legislative thinking, aiming to give full play to its specific functions through the introduction of the punitive damages system to better respond to social concerns and solve social anomie problems. ① To learn from other countries' systems, we need to trace the source of the system, explore the “growth environment” of the birthplace of the system, seek the purpose of establishing the system and summarize the practical effect, and then establish a punitive compensation system with Chinese characteristics in combination with the basic national conditions and the current situation of the rule of law. ② Whether punitive damages system can be applied in environmental public interest litigation. The judge made this judgment based on a series of circumstances in the case as a reference, which was a flagrant violation of civil liberties. ③ How to apply punitive damages system in environmental public interest litigation. The existing legal system lack legal provisions for the specific application of the punitive compensation system to environmental public interest litigation. How to ensure the implementation of the punitive compensation system in environmental public interest litigation, we need to solve the following four problems from the system: first, how to improve the distribution and standard of proof in litigation? Second, how can the punitive damages system avoid repeated abuse? Third, how to determine and dispose of punitive damages? Fourth, how does the plaintiff of environmental public interest litigation exercise the right to claim punitive damages?

## 5. Result Analysis

### 5.1. Improvement of the Burden of Proof and Standard of Proof of Punitive Damages

Punitive damages encourage the public to act as “private prosecutors” to achieve the function of the law to fill the damage, with the functions of punishing the defendant for malicious acts and deterring the defendant or others from engaging in similar illegal acts. For the infringed, there is no doubt that the punitive damages system is more “attractive.” The punitive compensation system enables the general public to exercise power on behalf of the national management subject and punish those who violate the provisions of the law. As the “agent manager,” the general public lacks supervision and management and cannot guarantee that the agent manager can still follow the basic principle of integrity and fairness of the civil law when exercising power. The punitive compensation system with the purpose of punishment and deterrence is opposed to the compensatory compensation system that restores the state before being infringed. Similar to the opposite relationship between criminal liability and civil liability, punitive compensation fittings have the nature of “quasi-criminal punishment” and should belong to the scope of criminal law or administrative law, but their nature is not completely the same as criminal fines or administrative fines. The former needs to be initiated by the infringed and is allowed to be withdrawn as a right, while the latter requires state organs to actively perform their duties according to the law and cannot be changed at will because of the clear provisions of the law. Due to the lack of supporting system, it is easy to blur the boundary between criminal law and civil law and it is easy to deviate from the original track. The application of punitive damages in the civil field lacks legal provisions for the procedural protection of infringers, especially the distribution of the burden of proof and the standard of evidence. The punishment of different cases is inconsistent (Table 1).

The calculation of departure from different security checks is as follows:

(3) $$\begin{array}{c} \text{Calculation of administrative penalty}:\text{final penalty method}=280000\text{ yuan}+\text{loss}\\ \text{expenses},\\ \text{Calculation of punitive damages}:\text{final penalty method}=\text{unit price of goods}\times 10\text{ times.} \end{array}$$

As for the burden of proof distribution of punitive damages, this involves two issues: one is whether the provision on the inversion of the burden of proof in article 1230 of the civil code is applicable to environmental public interest litigation, and the other is whether the inversion of the burden of proof rule is applicable to environmental public interest litigation, but whether the inversion of the burden of proof provision can be applied in punitive damages. Finally, based on the value orientation of the opposition between public law and private law, whether the proof of punitive damages in environmental public interest litigation should still apply the “high probability” proof standard of general civil cases, there are different views that the proof standard of punitive damages should be improved to ensure the legitimacy and rationality of punishment. From the perspective of infringers, environmental public interest litigation is different from criminal litigation or administrative litigation, and the latter two have reasonable protection procedures for infringers. In order to avoid the endless liability for compensation and the punishment of an “abnormal” amount for infringers, it is necessary to adjust the allocation of the burden of proof and the standard of proof in environmental public interest litigation. In addition, according to the persuasion of evidence, the litigation procedures are also different (Table 2).

### 5.2. Comparison between Punitive Compensation Liability and Criminal Liability

The nature and form of civil liability and criminal liability are inconsistent, which does not exclude the application. However, the punitive damages system, as the product of the development of public law of private law, is not a pure civil legal liability, which overlaps with the purpose of some types of punishment. As a punishment, its function is the same as that of a fine in criminal punishment, which reflects the economic punishment of infringers and can also serve as a warning to the society. The Supreme Court of the United States also has a special view on punitive damages. It believes that punitive damages are not compensation for damage, but a private fine imposed by the jury on the illegal actor to punish the defendant's conviction behavior. The fine is set to prevent the recurrence of similar behavior. ① The main purpose is to punish and sanction the behavior and subjective malice of the perpetrator. Therefore, punitive damages cannot compensate for the damage to the victim. In addition, some scholars believe that punitive compensation is a mixture of civil law and criminal law, and the punitive compensation system completes the deterrence purpose of criminal law. Therefore, the punitive compensation system has been criticized by some scholars as a “strange abnormal” or “abnormal” legal phenomenon, because the punitive compensation system injects the punishment and deterrence functions of criminal law into civil compensation, changing the coordination and scientificity of departmental laws. From the perspective of jurisprudence, criminal punishment is aimed at criminal acts, and punitive compensation is aimed at violations. In the relief procedure provided by the law, for criminal acts that affect public safety, the state, on behalf of the public, will impose various criminal punishments, such as public surveillance, criminal detention, fines, fixed-term imprisonment, life imprisonment, and even deprivation of political rights and the right to life, on the wrongdoers according to the criminal procedure. In the process of criminal punishment, the victim is only in the position of a private prosecutor or witness in the case of public prosecution. The effective judgment of the court does not directly care about the compensation of the victim, and the victim cannot get a realistic monetary remedy in the process of pursuing public law responsibility for criminal acts. The victim should first claim for the tort liability arising from the infringement to the court. The purpose of the lawsuit is to obtain compensation for the damage he suffered according to the implementation of the legal documents in force by the competent authority so as to fill the damage. As people usually understand it literally, punitive damages are born in addition to damages for the wrongdoer, to punish the wrongdoer for malicious or rude illegal acts, and to deter himself and others from similar illegal acts in the future. Although it is generally believed that the purpose of punitive damages is not compensation, and it is similar to criminal punishment, it is still quite different from criminal punishment (Table 3).

### 5.3. Determination, Attribution, and Distribution of Punitive Damages

At first, the purpose of applying punitive damages in the U.S. courts was to compensate for the losses of the infringed. Now, the purpose of punitive damages is more focused on punishing the infringer and deterring similar acts. From the perspective of compensation for the infringed to the “punishment” of the society for the infringer, the amount of punitive damages has also increased from dozens of dollars at the beginning to millions of dollars. Due to the emergence of some noteworthy “sky high” compensation, American academic circles began to criticize the punitive compensation system, pointing out that in a capitalist society, ordinary citizens have a natural resistance to large enterprises or companies, so it is difficult for the court to suppress their inner “indignation” during the trial. The application of punitive damages in infringement disputes should focus on the subjective malignancy of the infringement, rather than the severity of the damage results. However, due to the accusation of the infringed, the focus extends from the infringed to an unspecified third person, and the jury loses its reason and falls into the hypothetical coercion of the damage result. As a result, based on the unfortunate sympathy for the infringed and the moral disgust for the infringer, the punitive damages are not based on the justice standards or legal provisions of ordinary citizens, but on emotional trials, resulting in the uncertainty and unpredictability of the judgment results of the case. Compared with compensatory compensation for the purpose of compensation for damage, the purpose of punitive compensation is to punish the defendant for malicious illegal acts at the moral level. In fact, the punishment at the moral level is inseparable from the social acceptability standard of ordinary citizens for morality. The law cannot define the social standard for morality, but the law should limit the punishment standard, because the uncertain and unpredictable punitive damages have no fairness and justice, and the punitive damages obtained by the infringed lack legitimacy (see Table 4 for the details on the standard of compensation).

### 5.4. Establishment of Punitive Compensation Supporting Measures

On July 2, 2020, the procuratorate announced the relevant situation of the case and then filed a civil public interest lawsuit. However, on the day before the court session, it was temporarily decided to change the claim and require the defendant Hailan company to bear 171406.35 yuan of punitive damages for environmental infringement on the basis of the original claim. This measure is too sudden for both the defendant and the society. The application of punitive damages cannot only focus on “quantity” but ignore “quality.” Punitive compensation is for the needs of social public interest. As the plaintiff of environmental public interest litigation, the exercise of the right to claim punitive compensation should serve the social public interest and be supervised by the society. The “first cut and then play” litigation method is easy to make the punitive compensation system the “black box” of environmental public interest litigation. However, the existing announcement procedure is only to urge other organs and social organizations to file a lawsuit and will not affect the claims of public interest litigation.

## 6. Conclusion

Although the punitive damages system comes from foreign countries, it has gradually developed Chinese characteristics after nearly 30 years of practice in the judicial field in China. The system of punitive compensation for ecological environment is an important part of the tort liability of the civil code. It not only carries the burden of protecting the ecological environment of the civil code but also reflects the national policy of green development. However, it needs more in-depth research in the field of environmental public interest litigation. According to the argumentation of manager theory, it is suitable to institute punitive damages in environmental public interest litigation, which is helpful to realize the functional orientation of punitive damages. However, in the current judicial practice, it is still necessary to further improve the system and supporting measures for the application of punitive damages. At present, the urgent task is to further improve the standard of punitive damages through the introduction of judicial interpretation. At the same time, the burden of proof, standards of proof, and other relevant laws related to environmental public interest litigation should be adjusted to reduce the obstacles to the implementation of the punitive compensation system.

## Figures and Tables

**Figure 1:** Composition of sustainable development concept.

**Figure 2:** Framework of the civil code.

**Figure 3:** Public interest litigation.

**Figure 4:** Flowchart of civil public interest litigation.

**Figure 5:** Animal protection.

**Figure 6:** Defendant's response to the lawsuit in ecological infringement case.

**Figure 7:** Trial of civil infringement cases.

**Figure 8:** Ecosystem cycle.

**Figure 9:** Species data.

**Figure 10:** Schematic diagram of fault liability.

**Table 1:** Punishment of different types of cases.

Security check type	Illegal income	Penalty multiple
Administrative sanction	280000 yuan	2x
Punitive damages	280000 yuan	Up to 10 times

**Table 2:** Persuasion of evidence and litigation procedure.

Evidence	Proceedings	Plaintiff's ability to provide evidence
Clear and persuasive	Civil and criminal proceedings	Weak
Remove reasonable doubt	Criminal action	Strong
High probability	Civil action	Weak

**Table 3:** Comparison of different types of cases.

Type	Proceedings	Form of liability	Whether to allow abandonment
Punitive damages	Civil action	Civil	Allow
Fine	Criminal action	Criminal	Not allowed

**Table 4:** Compensation standard.

Compensation mode	Type of responsibility	Discretionary power	Operability
Fixed quota	Criminal fine liability	Lower	Low
Limit setting	Responsibility for administrative punishment	Higher	Higher
Unlimited amount	Responsibility for administrative punishment	Higher	Higher

## Data Availability

The labeled dataset used to support the findings of this study is available from the corresponding author upon request.

## References

[1] Zamula I., Prodanchuk M., Kovalchuk T., Kolesnikova O., Myhalkiv A. (2020). Indicators of ecological condition of natural resources in integrated reporting of the enterprise. *Naukovyi Visnyk Natsionalnoho Hirnychoho Universytetu*.

[2] Culp J. M., Brua R. B., Luiker E., Glozier N. E. (2020). Ecological causal assessment of benthic condition in the oil sands region, athabasca river, Canada. *Science of the Total Environment*.

[3] Shen Z., Zhang Q., Chen D., Singh V. P. (2021). Varying effects of mining development on ecological conditions and groundwater storage in dry region in inner Mongolia of China. *Journal of Hydrology*.

[4] Marín A. I., Abdul Malak D., Bastrup-Birk A., Chirici G., Barbati A., Kleeschulte S. (2021). Mapping forest condition in europe: methodological developments in support to forest biodiversity assessments. *Ecological Indicators*.

[5] Hanssen F., Barton D. N., Venter Z. S., Nowell M. S., Cimburova Z. (2021). Utilizing lidar data to map tree canopy for urban ecosystem extent and condition accounts in Oslo. *Ecological Indicators*.

[6] Shapiro A. C., Grantham H. S., Aguilar-Amuchastegui N. (2021). Forest condition in the Congo basin for the assessment of ecosystem conservation status. *Ecological Indicators*.

[7] Mayorova I., Temerbek A., Nosovckaj O., Ryabchuk V., Ocheredco E. (2021). Indicators of the seaport ecological state of a depressed industrial hub. *MATEC Web of Conferences*.

[8] Peszek Ł., Zgrundo A., Noga T. (2021). The influence of drought on diatom assemblages in a temperate climate zone: a case study from the Carpathian mountains, Poland. *Ecological Indicators*.

[9] Mukherjee K. (2020). Wetland habitat stability assessment in hydro-geomorphological (HGM) and surface water availability (SWA) conditions in a lower Gangetic floodplain region of eastern India. *Ecological Indicators*.

[10] Lam J. K., Cheung C. C., Chow M. Y. (2020). Transmucosal drug administration as an alternative route in palliative and end-of-life care during the covid-19 pandemic. *Advanced Drug Delivery Reviews*.

[11] Allen D. (2021). Using public interest litigation to achieve systemic change for people with a disability. *Australian Journal of Human Rights*.

[12] Jia X. (2022). On the sequence design and construction of the subject of environmental civil public interest litigation. *Modern Economics & Management Forum*.

[13] Rasquin C. (2021). Unlocking legal gridlock in high-income countries: how excessive litigation hampers growth and harms democracy. *Law and Development Review*.

[14] Durbach A., Reinecke I., Dargan L. (2021). Enabling democracy: the role of public interest litigation in sustaining and preserving the separation of powers. *Australian Journal of Human Rights*.

[15] Guo E., Jagota V., Makhatha M. E., Kumar P. (2021). Study on fault identification of mechanical dynamic nonlinear transmission system. *Nonlinear Engineering*.

[16] Huang R. (2015). *Framework for a smart adult education environment*.

[17] Liu J., Liu X., Chen J., Li X., Ma T., Zhong F. (2021). Investigation of ZrMnFe/sepiolite catalysts on toluene deg-radiation in a one-stage plasma-catalysis system. *Catalysts*.

[18] Ajay P., Nagaraj B., Pillai B. M., Suthakorn J., Bradha M. (2022). Intelligent ecofriendly transport management system based on iot in urban areas. *Environment, Development and Sustainability*.

[19] Sharma A., Rathee G., Kumar R. (2019). A secure, energy- and SLA-efficient (SESE) e-healthcare framework for quickest data transmission using cyber-physical system. *Sensors*.

[20] Jung J. A., Rogers H. N., Grabas G. P. (2020). Refinement of an index of ecological condition for marsh bird communities in lower great lakes coastal wetlands. *Ecological Indicators*.

